The article "Multiliteracies meet new methods: The case for digital writing in English education case study in G-7 countries" was retracted in 2025. Reasons: unreliable results or conclusions; concerns about the article.

# Multiliteracies meet new methods: The case for digital writing in English education case study in G-7 countries

**DOI:** 10.1371/journal.pone.0304343

**Published:** 2024-07-03

**Authors:** Xiaoying Hu

**Affiliations:** School of Foreign Languages, Inner Mongolia Minzu University, Tongliao, Inner Mongolia, China; Second Xiangya Hospital, Central South University, CHINA

## Abstract

Recently, globe has tried to transform populace activities to digital platform, wherefrom all stakeholders can attain their basic information. However, education sector cannot be excluded from this debate. Since, the pandemic mostly most economies have utilized digital transformation in different aspects of life, but digital education becomes more prominent. Therefore, this empirical research focuses on digital writing specifically to English education in G-7 economies between the time frame spanning from January 2000 to April 2022. This study considers urbanization, income, renewable energy, information & communication technology, renewable energy, English education, and pandemic as the key environmental determinants. To address the challenges posed by panel data, this study utilized an advanced set of estimators such as AMG stands for Augmented Mean Group. The estimate of urbanization and income per capita is positively significant, confirming that urbanization and economic development cannot protect the green economy by minimizing environmental pollution. Likewise, the estimated coefficient of English Education and internet use is negative and significant, implying that English Education and ICT can protect the green economy by reducing emissions. Conversely, renewable energy consumption (REC) is an element that can increase economic activity and therefore decline the environmental damages to secure a green economy. Likewise, the growth in cases of Covid-19 also reduces the usage of resources like land, water, and forests and subsequently decreases carbon emissions, promoting the green economy. The results also indicate that interaction term of English Education and ICT have adverse impact on Carbon emission (CO_2_). The outcomes suggest that internet usage (ICT) in English Education (EE) can deal efficiently with environmental issues for the green economy; therefore, EE and ICT should be part of green policies across the international level.

## 1. Introduction

The current climate change can be ascribed to the extensive use of environmentally harmful energy sources, especially fossil fuels. This alteration resulted in effects on both human and natural environmental conditions. If the ongoing rise in greenhouse gas (GHG) emissions persists, it will result in more warming and enduring alterations in all aspects of the climate system. The escalating rates of carbon dioxide (CO_2_) emissions have significant implications for both public health and environmental quality [1]. Numerous scientific fields have examined the detrimental impacts resulting from CO_2_ emissions. The academic and scientific researchers have focused on the topic of the effect of emissions on environmental quality [2]. The phenomenon of increasing sea levels and the persistent presence of global warming pose significant concerns. Nevertheless, the forecasts are even more unfavorable. As per a recent report conducted by the World Bank, it has been projected that global mean temperature will increase by 4°C compared to the pre-industrial period. According to Amanov et al. [3], it has been forecasted that heat extremes, sea-level rise, marine ecology, and water availability will reach a hazardous level in the near future. The scientific community has collectively identified greenhouse gas emissions as the primary driver of the observed global warming phenomenon. The main constituents of the greenhouse effect are water vapor, nitrous oxide (N2O), methane (CH4), and carbon dioxide (CO2). This has led to a rise in the average global temperature, resulting in climate change. Climate change presents a substantial threat to both human and ecological welfare due to its contribution to severe weather phenomena, an increase in sea levels, and the depletion of biodiversity [4].

Previous research on the role of higher education [5] in fostering the growth of a low-carbon economy has reached an advanced stage. The degree of education has a crucial role in promoting public consciousness regarding environmental conservation and fulfilling societal obligations [6]. Several scientists utilize CSS2013 data for their research, indicating a positive correlation between workers’ level of education and their adherence to environmental laws, rules, and obligations for environmental protection. In contrast to numerous academic areas, the field of English Language encompasses not only written academic English but also encompasses a broad range of English forms, such as oral English, informal English, and regional variations. The significance of this matter lies in the observation made by sustainability educator Chet Bowers, who highlights the interconnectedness between individuals and their surroundings in various social behaviors within local communities, hence fostering sustainability. Illustrative instances encompass social engagements centered on familial and social connections, communal engagement, admiration for the surrounding natural environment, artisanal pursuits, communal resource and labor sharing among neighbors, as well as local cultural festivities and commemorations [7]. The transmission of these traditions occurs through oral and informal means, and is transmitted intergenerationally via languages and dialects specific to the bioregion. Nevertheless, there is a prevailing inclination in the field of education to diminish the significance of particular local knowledge in favor of abstract, global, technical, and academic information. Nevertheless, it is worth noting that educational achievement has the potential to contribute to environmental deterioration by fostering the growth of endeavors that need a lot of energy, for instance manufacturing and transportation, while also facilitating the adoption of environmentally harmful technologies, such as vehicles [8]. English Education, despite its significant role in fostering human capital and clean technology, is not regarded as a determining factor for CO_2_ emissions. As far as the writers are aware, the sole study that has investigated the correlation among English Education (EE) and environmental quality is referenced. Their claim is that a prospective increase in energy consumption can result from the growth of both industries and urban areas. Within this framework, the authors highlighted the fact that English Education has evolved into a sector that applies universally. They emphasized that the construction of new buildings, dorms, and facilities to accommodate students will result in an increase in CO_2_ emissions due to the generation of ENE. Without a doubt, the growth and advancement of English Education can significantly impact CO_2_ emissions. However, the impact of positive externality created by English Education on the environment was overlooked by Simamora et al. [9]. The acquisition of knowledge, information, and skills has emerged as pivotal elements that define contemporary society, particularly in the latter part of the twentieth century.

A further strategy for mitigating CO_2_ emissions is leveraging ICT to circumvent the need for transportation, hence leading to a reduction in pollution levels. The European Commission’s assessment indicates that the internet has the potential to boost energy efficacy, which ultimately lead to a reduction in usage of energy and a favorable influence on ecological quality. The progress of ICT has been rapid over the past two decades. Several nations are keen in acquiring knowledge on leveraging information technology to reduce energy consumption and mitigate environmental harm. Previous empirical study has identified the utilization of information technology as a viable strategy for enhancing economic growth by simultaneously improving efficiency and reducing energy consumption. ICT has the potential to enhance productivity in production and decrease the consumption of material goods, leading to a reduction in energy demand and therefore alleviating the environmental impact [10]. ICT additionally aids in reducing paperwork, thereby exerting a favorable impact on environmental quality. ICT-focused strategies, such as videoconferencing or integrated point-of-sale systems, can reduce the environmental impact of enterprises. Nevertheless, the growing prevalence of e-learning has resulted in a decrease in travel, hence exerting a detrimental impact on CO_2_ emissions. The effect of internet usage on CO2 emissions, whether beneficial or detrimental, requires the proper execution of its function. The fundamental effect of the internet on fiscal activities lies in the transformative impact on production technologies and the introduction of a knowledge-intensive production model. The aforementioned features impose elevated standards on the caliber of the workforce. Advanced human capital often possesses a greater ability to allocate production factors, innovate technologically, and absorb knowledge. Enhancing human capital levels will amplify the beneficial effects of internet usage on manufacturing development and the reduction of CO_2_ emissions [11]. The attainment of sustainable usage of natural resources is unattainable in the presence of an ignorant labor force [12]. The technological spillover benefits of the internet are significantly limited in regions with lower levels of education due to their inadequate information digestion and technology conversion capacities, despite the potential for the internet to deliver the same knowledge stock [13].

The ongoing COVID-19 epidemic is leading to significant changes in all aspects of social, labor, political, and economic life. Various governmental bodies have implemented emergency policy measures, such as the postponement of classes and the closure of educational institutions, in order to remotely conduct teaching activities from homes using ICTs. This approach aims to mitigate the spread of infections [14]. The primary goal of this research was to measure the ramifications of the epidemic within the realm of education. In the framework of the paradigm shift from on-campus teaching to online teaching, education experts are confronted with the challenge of adapting to the new worldwide context facilitated by the online modality. This movement has been and continues to be characterized by its rapid and abrupt nature. The provision of quality education is contingent upon the advancement of information technology in various aspects, including enhancing learner motivation, enriching fundamental abilities, and augmenting teacher training in technology. The ICT is utilized as a tool for curriculum and subject transformation, effectively employed to establish a learner-centered environment. Teachers utilize ICTs to facilitate the acquisition and utilization of innovative pedagogical approaches by pupils. ICTs are becoming an essential component of the education system. It has significantly altered various facets of individuals’ life. The aforementioned changes have prompted educational institutions, administrators, and teachers to reconsider their responsibilities, teaching methods, and future vision. The field of ICT has faced new obstacles in ensuring high-quality education for learners. According to the Musah et al.[15], ICTs have the ability to enhance access to education and improve its relevance and quality in developing nations. The ICTs play a significant role in facilitating the acquisition and assimilation of knowledge. This presents developing nations with unparalleled prospects to better their educational systems, refine policy development and implementation, and expand chances for business and those living in poverty. The integration and utilization of educational technology into the educational systems of developing nations have encountered numerous challenges and do not consistently yield commensurate enhancements in student learning achievements. Therefore, it is crucial to undertake a comprehensive analysis and understanding of the key determinants of success in order to optimize student achievements through the utilization of ICT and digital learning tools inside higher education institutions [16]. The interconnection between higher education and sustainability is well recognized in contemporary society. In contemporary society, higher education bears the obligation and plays a crucial role in redefining education to promote sustainability, alongside its traditional responsibilities of doing research and delivering instruction. Conversely, technology has significantly facilitated the accessibility of resources for individuals both domestically and internationally. The expansion of technology-assisted learning has been occurring at a rapid pace [17]. According to the Lu et al. [18], the objective of education pertaining to sustainable development is to motivate learners and individuals they impact to embrace sustainable practices. The global adoption of ICT has increased due to reduced costs of computer technology, enhanced Internet access, and improved digital infrastructure in many countries. However, it was initially mentioned that digital learning provides the less developed globe with a chance to expand education and ensure equitable access to education at reduced costs [19]. Consequently, they play a crucial role in digital learning for sustained development [20]. The correlation between the utilization of ICT and the academic achievement of students in higher education remains ambiguous, with current research yielding conflicting results. A prior investigation has been unable to arrive at a definitive determination regarding the influence on student achievement [21].

This study provides three notable contributions to the current corpus of academic research. This research is a limited exploration of the determinants that impact GDP per capita, English Education (EE), and ICT within the G-7 nations. The G-7 (group of seven) consists of the most advanced industrialized nations worldwide namely Germany, France, Italy, Japan, Canada, the United Kingdom, and the United States of America. Despite comprising only 11% of the global population, the G-7 has a significant proportion of the world’s economic output, up to 33% when balanced for purchasing power. This highlights its crucial role in the global economy. These seven countries collectively account for 33% of the world economic output. Despite the prevailing economic slump, a significant number of the G-7 nations have effectively enhanced their economic performance in real terms in past years. Notably, the United States and Canada have witnessed the most significant increases in their Gross Domestic Product (GDP). The outcomes of our study will provide significant perspectives for representatives in formulating and executing health and education programs. The second aspect of our study is to the range of indicators utilized. There exists a considerable body of literature examining the relationship between GDP per capita, urbanization, English Education, ICT, renewable energy, and COVID-19. However, there is a scarcity of studies that specifically investigate the impact of these factors on the sustainable environment within the G-7 region. This research contributes to the current knowledge by providing experiential evidence on the influence of GDP per capita, urbanization, English Education, COVID-19, renewable energy, and ICT on CO_2_ emissions in the G-7 countries. The present analysis additionally demonstrates the moderating influence of English Education and ICTs on CO_2_ emissions in G-7 economies. However, previous scholarly research has examined the aforementioned correlation. However, the contradictory results indicate a vague understanding of the correlation among developing nations. Therefore, this study offers a precise portrayal of the aforementioned link in developing economies. The long-term dynamics of G-7 are analyzed through the application of scientific and empirical approaches. The research employed contemporary econometric methodologies, including second-generation panel unit-root [22], the cross-sectional dependency test, and second-generation cointegration tests [23]. Additionally, Augmented Mean Group (AMG) approaches were utilized for lung run estimate. The main aim of this study is to clarify the associations between GDP per capita, urbanization, English Education, ICT, renewable energy, and the effect of COVID-19 on ecological deterioration, specifically in respect to CO_2_ emissions.

The following sections of this work are organized as follows: The section on "Literature review" evaluates the existing literature, the section on "Methodology and data" provides a summary of the methodology employed, and the section on "Empirical results & Discussion" examines the data and deliberates on the main conclusions. The concluding section of the study presents a summary and provides policy suggestions.

## 2. Literature review

### 2.1. Education and carbon emission (CO_2_)

The existing literature presents comparable findings about the significance and advantages of education in mitigating carbon emissions and attaining ecological footprints [24,25]. The aforementioned circumstances have prompted a demand for the advancement of sustainability education within institutions of advanced education and the business sector, with the aim of mitigating greenhouse gas emissions [26]. This encompasses the promotion of online education, as evidenced by the works of Meissner et al. [27]. Multiple studies have shown evidence for the positive influence of education on environmental sustainability. These studies have recommended that more resources be allocated to education in order to improve ecological quality [28]. Naor et al. [29] argue that education remains highly significant at both the individual and national levels. This is because improving educational levels aligns with the Sustainable Development Goals (SDGs) [30].

Higher education is closely connected to sustainable development [31]. In a study conducted by Amanov et al. [3], it was shown that there is a notable influence of the scale and caliber of higher education on carbon emissions. The researchers analyzed panel data from 31 provinces in China and observed that an expansion in both the size and quality of higher education institutions leads to a decrease in carbon emissions per person. In their study, Elbes et al. [4] analyzed the greenhouse gas emissions composition at Yale University and delineated the influence of university behavior on carbon emissions. Higher education plays a crucial role in driving technological advancements, which in turn contribute significantly to industrial transformation. These advancements have the potential to enhance the energy utilization structure and improve energy efficiency effectively [32].

Nevertheless, the enduring consequences of this phenomena are both positive and significant. These findings indicate that in order to impact the economy, policies and reforms pertaining to the educational system, as well as measures to decrease carbon emissions and address climate change, must have lasting consequences [33]. Therefore, directing resources towards education, particularly in impoverished countries, has the potential to result in significant and long-lasting effects in terms of reducing carbon emissions and addressing the challenges posed by climate change.

While the literature explores several factors related to the main causes of CO_2_, the potential effects of EDU on ecological degradation have not captured the attention of academics. EDU can have both good and bad effects on CO_2_ through many processes. The research carried out by Sart et al. [34] assessed the association between economic freedom, EDU, and CO_2_ emissions within the European Union (EU) member states from 2000 to 2018. The analysis of causality indicated that financial freedom and education have the potential to support positively to the mitigation of environmental degradation and the enhancement of ecological quality within the chosen panel region. Therefore, it is imperative to acknowledge the enduring impacts of education, as it fosters heightened social and cultural consciousness and accountability [35]. The study done by Lee et al. [36] observed the influence of education on the climate in 22 developing countries between 1990 and 2016, employing the ARDL approach. They discovered that, above a certain degree of educational achievement, the substantial influence of poverty on climate change can decrease. Additionally, some recent research looks at the direct connection between pollution discharges and environmental deterioration and education [37,38]. As a result, since they support renewable energy, human resources, physical education, and educational status all help to construct the EKC and reduce air pollution.

### 2.2. ICT and carbon emission (CO_2_)

ICT abbreviation of Information and Communication Technology is generally recognized as a significant driver of economic growth on a global scale. The negative impact of energy utilization and internet usage have been reaffirmed in recent research conducted by Wang et al. [39]. These studies collectively conclude that the increasing prevalence of internet usage has harmful effects on the environment because of its high energy consumption. Adebayo et al. [40] examined the causal relationships, both in the short-run and long-run, among energy utilization, CO_2_ emissions, economic growth, and information and communication technology (ICT) across several financial sectors in Iran during the period of 2002 to 2013. In their study, Xie et al. [41] employed fixed effects and quantile regressions to examine the 13 chosen G-20 countries. Their findings did not provide evidence in favor of the EKC. Nevertheless, the researchers did demonstrate that ICT, trade openness, and technology have a role in mitigating emissions. Laddha et al. [42] analyze the association between ICT, trade globalization, and carbon emissions in six Association of Southeast Nations. They employ panel cointegration techniques and observe that both ICT and trade globalization have a negative effect on CO_2_ emissions. In their study, Wendt et al. [43] examine the influence of ICT in four Sub-Saharan African nations and three East Asian and Pacific countries. Their findings indicate that the influence of ICT varies among the countries under investigation. In their study, Chatti et al. [44] examine the association between industrial structure, urbanization, and emissions in South Africa over a span of four decades (1975–2014). Their results indicate an adverse impact of manufacturing production on carbon emissions, but urbanization has an opposing effect. Erumban et al. [45] conducted a research, in this research an examination was undertaken on 10 Asian countries spanning the years 1994 to 2019. The findings of the study indicate that the utilization of ICT has a beneficial effect on environmental quality. The study explores the correlation between CO_2_ emissions, ICT and financial development by constructing a panel consisting of nine ASEAN countries spanning the years 1991 to 2009. Rehman et al. [46] has identified a significant positive correlation between ICT, economic growth, and CO_2_ emissions.

Numerous experts direct their study towards examining the economic ramifications of digitization. Certain scholars argue that digitalization has the potential to enhance employment efficiency, facilitate advancements in industrial structure, reduce income inequality, and influence urban spatial patterns through the optimization of factor resource allocation [47]. Nevertheless, there is an incomplete body of study that specifically emphases on the correlation between digitization and haze pollution. The majority of research endeavors primarily focus on investigating the causal connection between ICT and CO_2_ emissions. However, there exists a lack of agreement regarding the efficacy of ICT in mitigating carbon emissions. Some scholars contend that the use and progress of information and communication technology (ICT) not only promote the development of ecologically sustainable and low-carbon lifestyles among individuals [36], but also empower businesses to participate in intelligent sustainable production and management of energy. This, in turn, fosters innovation in green public welfare and service provision, resulting in a dual enhancement of production competence and carbon competence. Consequently, ICT progressively emerges as a potent catalyst for the transition towards low-carbon practices [48]. However, it has been argued by other scholars that the process of digitization presents both potential and significant obstacles in the context of haze pollution control [35]. During the early phase of digitalization, the proliferation and widespread use of ICT goods have resulted in heightened energy consumption and environmental degradation [49]. In previous years, there has been a significant rise in energy consumption resulting from the use of ICT products, with an annual growth rate of 7% [50]. Wang et al. [51] reported that the global energy consumption caused by the utilization of ICT-related items has risen to 4.7% by 2012, indicating a 3.9% increase compared to 2007.

### 2.3. ICT and education

Dadashpoor et al. [51] Similarly, the aforementioned remark is reiterated, with the inclusion that the primary objective of a class is for instructors to accomplish their objectives. Consequently, the utilization of ICT is often limited to pupils carrying out tasks as instructed by the teacher. According to **Nair et al.** [52], ICT is seldom used as a means of communication between instructors and students. This circumstance exemplifies the promotion of ICT in education without enough attention to pedagogical concerns, resulting in the use of ICT becoming a goal in itself rather than a means to enhance teaching and learning effectiveness. The initial investigation [53] and subsequent study done by Huang et al. [54] exposed that the utilization of ICT in educational endeavors is a subject that has received insufficient attention in the Nepalese context, and there is a scarcity of literature available in this domain. Nevertheless, research indicates that this is an extensively studied field, especially in industrialized nations, particularly those in the western hemisphere. Adarkwah et al. [55] examined the observations and motivations of pre-service teachers and discovered that they had a commendable level of awareness and enthusiasm for using ICT into educational practices. However, a limited number of difficulties were detected regarding the facilities and technical expertise. The objective of this study was to begin the process of establishing a professional growth program that would be most advantageous to the faculty at this Higher Education Institution (HEI). The study was carried out at the College of Education [56], which is the highest-ranking institution for teacher training in Liberia. The research was designed to investigate the challenges associated with the integration of ICT in teachers’ education, provide strategies to mitigate these challenges, and ultimately enhance the overall integration process.

In addition, the incorporation of ICT into education is intricately linked to the decision-making process of educators who serve as leaders in implementing educational practices [57]. Educators must possess extensive knowledge of the capabilities of different types of ICT and be skilled in determining the optimal timing, methods, rationale, and specific technologies that will yield the greatest benefits for classroom instruction [58]. Insufficient understanding of ICT integration can result in improper utilization, which in turn leads to children having passive roles and insufficient guidance in their replies [59]. As a result, this condition may provoke adverse feelings in youngsters and restrict their chances for learning [60]. The concern regarding inappropriate usage not only endangers the educational advantages of ICT but also increases the likelihood of educators completely avoiding its use.

## 3. Data and methods

This empirical research tries to introduce an innovative series of environmental determinants under the current scenario of pandemic in G-7 economies over the period of January 2020 to April 2022. However, these determinants are income urbanization, ICT, renewable energy, English education and Covid-19. The selected of variables has been made on two logics; firstly, the pandemic situation immensely has disturbed all the human & economic activities. Secondly, education sector has more influenced from the pandemic; therefore, economic have tried their best to shift the physical education system to online with the help of digitalization. Thus, English education entirely dependent on the digitalization. However, selected variables units, sources and symbol are detailed in Table 1.

**Table 1:** Description of variables.

Symbol	Unit	Sources
CO_2_	Carbon emissions (KT)	WDI
GDPC	Income per capita (Current US$)	WDI
URB	Urbanization (% of total population)	WDI
ICT	Information & communication technology (Individuals using the Internet, % of population)	WDI
RE	Renewable energy consumption (% of total energy consumption)	WDI
EE	English education (# of students in English taught education)	MRD
Covid-19	deaths per million people	OWD

Note: OWD: Our world in data, WDI: World bank development indicators.

**Ethical Approval and Consent to Participate**: The authors declare that they have no known competing financial interests or personal relationships that seem to affect the work reported in this article. We declare that we have no human participants, human data or human tissues.

### 3.1. Theoretical background

Ehrlich and Holden created the IPAT identity in the early 1970s [61] and it has since been accepted as a conceptual framework for examining human-caused environmental change. There are three drivers of environmental impacts in the IPAT model: population, prosperity, and technological advancements. It is possible to express the IPAT model as follows:

I=P×A×T (1)

There are several limitations to the ImPACT and IPAT models since they do not allow the influencing factors to varying non-monotonically or in proportion to each other. These researchers reworked IPAT’s identity into a stochastic form (STIRPAT) to overcome this issue, creating the STIRPAT model. Environmental change can be studied by using this stochastic model, which is commonly used to investigate the impact of driving forces. It’s possible to express the STIRPAT model mathematically as follows:

$${\text{I}}_{\text{i}}=\alpha \cdot {\text{P}}_{i}^{b}\cdot {\text{A}}_{i}^{c}\cdot {\text{T}}_{i}^{d}\cdot {\text{e}}_{\text{i}}$$ (2)

the model’s constant coefficient is a, while the underestimated parameters are denoted by b, c, and d, with the error term denoting e. A, B, C, D, and E are all equal to 1, which means that the IPAT model will be used instead of the IPAT model. It is possible to change Eq (3) into: after taking the log.


$$\ln\;{\text{I}}_{\text{i}}=\ln\alpha +\text{b}\;\ln\;{\text{P}}_{\text{i}}+\ln\;{\text{A}}_{\text{i}}+\ln\;{\text{T}}_{\text{i}}+\ln\;{\text{e}}_{\text{i}}$$ (3)

Understanding the dynamic interactions between human systems and the environments on which they depend is the goal of IPAT/STIRPAT. Each coefficient in the STIRPAT model can be estimated as a parameter, and the proper decomposition of each element is possible. Thus, new influencing factors can be introduced to the STIRPAT model context as said by the specifics of each study. The STIRPAT model examines ecological change from both a technical and policy perspective. The IPAT/STIRPAT model is now the most widely utilized and renowned theoretical framework for examining the influence of CO_2_ emissions on the atmosphere. The STIRPAT theoretical model is extended based on earlier research to fulfill our design needs.

The primary motivation for developing the initial extension was the association between the efficiency of fossil fuels and CO_2_ emissions. Fossil energy efficiency measures how effectively a production process utilizes fossil energy compared to the useful output that results from that process. Furthermore, this research investigates the proportion of REC in the energy composition, which has the capacity to lessen CO_2_ emissions by diminishing the direct utilization of fossil fuels. It also incorporates the concept of "human capital," which refers to a person’s English education level. This was followed by the Covid-19 case, expressed as a decline in the proportion of positive patients throughout the provinces as a rationale for steady reductions in carbon emissions. Urbanization and economic advancement in terms of Per capita income, which can explain exogenous increases in CO_2_ emissions that are not defined by other independent factors, were also incorporated. The World Health Organization and the World Development Indicator (WDI) provided all the information.

A dynamic panel data model based on this information is proposed:

$${\text{LCO}}_{2\;\text{I,t}}+\beta_{0}{+\beta }_{1}{\text{lnURB}}_{\text{i,t}}{+\beta }_{2}{\text{lnGDPC}}_{\text{i,t}}{+\beta }_{3}{\text{lnICT}}_{\text{i,t}}{+\beta }_{4}{\text{lnEE}}_{\text{i,t}}{+\beta }_{5}{\text{lnRE}}_{\text{i.t}}{+\beta }_{6}{\text{lnCovid}}_{\text{i.t}}{+\mu }_{\text{i.t}}$$ (4)

Here, i is the country, and t is the year, and CO_2it_ is the total amount of CO_2_ emitted by specific provinces I throughout the year; Urbanization is referred to as URB. Economic output per capita is referred to as GDPPC; ICT reflects the number of internet users per person. β1-β6 are estimated parameters, whereas I as a random disturbance term. EE shows the symbol of English education. RE denotes the fraction of REC. The World Health Organization and World Bank provided all of the data used in the study.

However, an additional aim of this research is to examine the mild impact of English Education and Information and Communication Technology (ICT) on carbon emissions (CO_2_). Likewise, the moderate effect Eq 5 are inserted below:

$${\text{LCO}}_{2\;\text{I,t}}=\beta_{0}{+\beta }_{1}\;{\text{lnURB}}_{\text{i,t}}{+\beta }_{2}\;{\text{lnGDPC}}_{\text{i,t}}{+\beta }_{3}\;{\text{lnICT}}_{\text{i,t}}{+\beta }_{4}\;{\text{lnEE}}_{\text{i,t}}{+\beta }_{5}\;{\text{lnRE}}_{\text{i.t}}{+\beta }_{6}\;{\text{lnCovid}}_{\text{i.t}}{+\beta }_{7}\;\left({\text{lnEE}}_{\text{i,t}}{*\text{lnICT}}_{\text{i,t}}\right){+\mu }_{\text{i.t}}$$ (5)

In the subsequent model, we add the association term between English Education and information & communication technology (lnEE_i,t_ * lnICT_i,t_). The β7 represents the coefficient of the interaction term.

### 3.2. Estimation strategy

In panel data, overlooking the CSD can lead to major problems. Three tests are used to conclude the best panel technique, including [62,63]’s CSD test. The mathematical form of the CSD ratio test can be presented as follows:

The form of the CSD ratio test can be described as follows,

$$\text{CD}=\sqrt{2T/N(N-1)}\left(\sum_{i=1}^{N-1}\sum_{j=i+1}^{N}\rho ij\right)\;N(0,1)$$ (6)

$$\text{FRI}=(\text{T}-1)\left[\frac{2}{N}\sum_{i=1}^{N-1}\sum_{j=i+1}^{N}\gamma ij+1\right]\;\chi^{2}(\text{T}-1)$$ (7)

$$FRE=\frac{(\text{T}-1)\left[\frac{2}{N}\sum_{i=1}^{N-1}\sum_{j=i+1}^{N}\gamma ij+\frac{1}{T}\right]}{SE(Q)}\;\text{N}(0,1)$$ (8)

Here, the coefficient of residual association from individual OLS regression is utilized. ij denotes the estimated value of the Spearman’s rank coefficient, whereas SE (Q) represents the standard error of the Q distribution. The formulation of Fisher’s initial unit root test when using Panel CSD is as follows:

$${\Delta \text{y}}_{\text{i},\text{t}}=\alpha_{\text{i}}+\gamma_{\text{i}}{\text{y}}_{\text{i},\text{t}-1}+\sum_{j=1}^{k}\alpha jyi,t-1+\varepsilon_{\text{j},\text{t}}$$ (9)

The term Δyi,t is used to indicate the random disturbance term, which is the first difference between yi and T at the i-th observation of the panel. This term is comparable to γ, εi, and t. The utilization of CADF as the second-generation unit root test has been documented by Pesaran et al. [64].


$$\Delta {\text{y}}_{\text{i,t}}=\alpha_{\text{i}}+\beta_{\text{i}}*{\text{y}}_{\text{i,t-1}}+{\text{d}}_{0}{\text{y}}_{\text{t-1}}+\sum_{j=0}^{p}d\;j+1\Delta {\text{y}}_{\text{i,t-j}}+\sum_{k=1}^{p}Ck\;\Delta {\text{y}}_{\text{i,t-k}}+\mu_{\text{i,t}}$$ (10)

Using the CADF model, the mean of the t statistics of the parameter β* can be used to approximation CIPS.


$$\text{CIPS}=\sum_{i=1}^{N}\;\frac{t}{N}$$ (11)

Co-integration testing is the following step. When both series are listed in the same order, an association between concern variables is formed. It is possible to discover long-term equilibrium processes with the help of a handy technique called co-integration. The Durbin Hausman group men co-integration test, which was developed by [65], was utilized by our team. Additionally, prior acquaintance with the integration sequence of variables is not required for this test because the CD ratio is applicable in this particular test. In light of this, it is something that can be applied in the future conditions.

### 3.3. Augmented mean group and long-term association

Panel estimators may yield inaccurate, subpar, and sometimes inconsistent estimates when models are affected by contemporaneous dependence (CD), heteroskedasticity, and serial correlation [64]. These challenges have been alleviated by Pesaran [65] proposal of the Common Correlated Effects [66]. This methodology offers notable improvements as compared to the initial generation of econometric techniques. It does not take into account any common factors that have not been unnoticed and factor loadings [67]. We will use the Augmented Mean Group (AMG) algorithm [68] in this part of our research. The AMG model may effectively accommodate time-varying variables while estimating parameters, without any limitations [69]. Below is a diagram of the main panel model.


$${\text{lnCO}}_{2\;I,t}=\beta_{0}+\beta_{1}\;{\text{lnURB}}_{\text{i,t}}+\beta_{2}\;{\text{lnGDPC}}_{\text{i,t}}+\beta_{3}\;{\text{lnICT}}_{\text{i,t}}+\beta_{4}\;{\text{lnEE}}_{\text{i,t}}+\beta_{5}\;{\text{lnRE}}_{\text{i.t}}+\beta_{6}\;{\text{lnCovid}}_{\text{i.t}}+\mu_{\text{i.t}}$$ (12)

The first differenced form of the aforementioned equation yields the following results:

$$\text{lnCO2}\;\text{I,t}=\beta 0+\beta 1\;\text{lnURBi,t}+\beta 2\;\text{lnGDPCi,t}+\beta 3\;\text{lnICTi,t}+\beta 4\;\text{lnEEi,t}+\beta 5\;\text{lnREi.t}+\beta 6\;\text{lnCovidi.t}+\sum_{t=2}^{T}pt(ADt)+\mu_{\text{it}}$$ (13)

In the case of T-1 period dummies, ADt refers to the initial difference; in this case, pt refers to the parameters. ADt the assessed parameter pt is replaced with T variables in the following phase, which indicates the dynamic technique as follows:

$$\text{lnCO2}\;\text{I,t}=\beta 0+\beta 1\;\text{lnURBi,t}+\beta 2\;\text{lnGDPCi,t}+\beta 3\;\text{lnICTi,t}+\beta 4\;\text{lnEEi,t}+\beta 5\;\text{lnREi.t}+\beta 6\;\text{lnCovidi.t}+d_{1}\left(\delta_{\text{t}}\right){+\mu }_{\text{it}}$$ (14)

$$\text{lnCO2}\;\text{I,t}-\delta_{\text{t}}=\beta 0+\beta 1\;\text{lnURBi,t}+\beta 2\;\text{lnGDPCi,t}+\beta 3\;\text{lnICTi,t}+\beta 4\;\text{lnEEi,t}+\beta 5\;\text{lnREi.t}+\beta 6\;\text{lnCovidi.t}+\mu_{\text{it}}$$ (15)

### 3.4. D-H panel causality test

Additionally, we use the Dumitrescu-Hurlin (D-H) panel Granger causality test [70], which allows us to capture the grade of heterogeneity across each given country, to investigate the relationships between the variables. It is Granger’s non-causality heterogeneous panel data test that is the foundation of the D-H panel Granger causality test. For every panel cross-section, the homogeneously non-causality null hypothesis states that the variables do not have any causal relationship with one another. Standardized mean average Wald statistics, for example, are simple to compute and follow a standardized asymptotic normal distribution; this is the main benefit of this method;

HNC abbreviated as the null Homogenous Non-Causality hypothesis is known to be associated with the average statistic $W_{N,T}^{H_{nc}}.$


$$W_{N,T}^{H_{nc}}=\frac{1}{N}\sum_{i=1}^{N}W_{i,T},$$

The individual Wald statistics for the *i*th " cross-section unit according to the individual test *H*_0_ = *β*_*i*_ = 0 were denoted by *W*_*i*,*T*_.

IRF and variance decomposition outcomes are included in the results, as well. Fig 1 displays a scatter plot of the variables.

**Fig 1:** Scattered plot of the used variables.

## 4. Results and discussion

Table 1 demonstrate the statistical explanation of the selected variables. So as to guide future empirical research. This study focuses on the green economy (CO_2_ emissions), urbanization, income per capita, renewable energy consumption, ICT, English Education, and Covid-19 cases. Table 2 demonstrates that there is no significant difference between the median and mean values.

**Table 2:** Descriptive statistics of the variable.

Variable	lnCO_2_	lnURB	lnGDPC	lnICT	lnEE	lnRE	lnCOV-19
Mean	0.7083	5.8963	4.7712	8.4402	4.5623	7.2456	0.9632
Median	0.7033	5.6624	4.3412	8.1289	4.0874	7.1274	0.8819
Minimum	0.0456	1.7452	0.4523	1.5241	0.2289	1.3334	0.0024
Maximum	3.7895	9.5235	8.2469	14.5621	7.3345	11.9642	1.6578
Standered Deviation.	00.3124	00.8923	00.0127	00.2354	00.3425	00.8942	00.1245
P-value	0.001	0.004	0.002	0.001	0.001	0.002	0.0001

We begin our study using the cointegration tests and unit root that best match our data. As previously mentioned, the study makes use of a variety of CD ratio tests. Results of CD tests in various provinces are given in Table 3. Can be seen in table all of these test’s discard H0 of CD statistically at the 1% significance level. Hence CD is included in each series.

**Table 3:** CDs test.

Test	Value	P-value
CD	30.971	0.003
Q	9.6341	00.001
CD	265.342	0.005

The results of the unit root tests are motioned in Table 4. The findings of the CADF tests demonstrate that carbon emissions and English Education are static at the level, while URB, GDPC, RE, ICT, and Covid-19 are static at the first difference for the economies tested.

**Table 4:** CADF unit root test.

Variable	CADF	
	Level	1st difference
lnCO_2_	-2.091*	-5.335*
lnURB	-1.985	-4.238*
lnGDPC	-1.136	-5.976*
lnEE	-3.572*	-7.914
lnICT	-1.853	-4.102*
lnRE	-1.134	-3.892*
lnCovid	-1.945	-6.329*

Before looking at long-term correlations between variables, it is important to identify the unit root. This is accomplished using a cointegration test with error correction suggested by [71]. The term negative error correction is a sign of cointegration’s prevalence. Several factors make the test appropriate for use in this investigation. First and foremost, it permits a high grade of heterogeneity in terms of short-term dynamics and long-term cointegration [72]. Second, it’s conceivable that the CD is behind it. Thirdly, the bootstrap options available in this test allow for numerous runs of the cointegration test to be conducted. Gt and Ga (group means tests) were used .H1 indicates that the panel is cointegrated in the test’s Pt and Pa. With regard to income strata, it was found that the no-panel cointegration hypothesis could not be refuted by Westerlund et al. [73], Gt and Ga, or Pt and Pa test statistics. Another way of putting it is that concern has a long-term association with the variables studied. Table 5 also discusses Westerlund’s findings.

**Table 5:** Westerlund cointegration test.

Statistics	Value	Z-value	P-Value	Robust P-Value
G_t_	-9.254	6.441	1.004	0.003
G_a_	4.324	7.245	1.000	0.554
P_t_	-1.995	5.882	1.000	0.099
P_a_	-7.582	3.445	1.000	0.005

### 4.1. Results of augmented mean group

According to this study, the digital economy, English education play a significant role in the green economy. Accordingly, the purpose of this research is for G-7 countries to better comprehend the impact of economic and urbanization growth as they relate to green economy features such as English Education, RE consumption, and the Covid-19 case studies discussed earlier this year. Primarily, urbanization positively impacts carbon emissions in the locations investigated. According to the study’s conclusions, one percent more urbanization in G-7 countries might lower carbon emissions by 0.634 percent. Purnamawati et al. [74] and Saha et al. [75] discovered that If environmental policies from industrialized countries can be implemented successfully in G-7 countries, then this could explain why the country’s ecology is degrading as a result of urbanization. Acts such as these, coordinate and harmonize environmental pollution control legislation, provide for environmentally-friendly management of natural resources, and further related goals. G-7’s government enacted and revised this law to protect the environment while enforcing heavy penalties against anyone who violates it. According to Alola et al. [76], the combination of high income and energy-intensive lifestyles among urban populations leads to a notable increase in greenhouse gas (GHG) emissions. Consequently, there is a greater need for urban transportation. Consequently, the development of public transportation infrastructure in metropolitan regions is undertaken to meet the escalating demand, thereby resulting in a rise in car ownership and subsequent escalation in road energy consumption. In the absence of an efficient and environmentally friendly public transportation infrastructure, unplanned urbanization leads to a rise in energy utilization by automobiles and GHG emissions. The present research yields result that align with the findings of [17,20,24], who conducted investigations on the correlation between urbanization and environmental quality across various geographical locations or regions.

It is also worth noting that real per capita GDP is significant at the one percent level, which means the level of carbon emissions might rise by 0.540 percentage points if real per capita GDP increased by one percent. It is therefore linked to additional environmental degradation as a result of its direct effect on carbon emissions. Increased machinery usage, particularly in the industrial sector, is necessary for economic expansion. As a result, more carbon emissions are produced, which can damage the immediate environment. As an outcome, improved economic activity encourages the deterioration of environmental conditions. According to F. Wang et al. [77] for European countries, this conclusion is in accordance with previous research. Studies have revealed that a reduction in carbon emissions would have a negative effect on financial development around the world [78]. Moreover, Guo et al. [79] found that increased carbon emissions lead to higher economic growth. In contrast to what Z. Wang et al. [80] observed, carbon emissions in Asia did not lead to economic growth.

Both internet penetration and carbon emissions have a negative impact on ICT variables, which are considered at the 1% level. In other words, more people having access to the Internet mean less CO_2_ being emitted into the atmosphere. ICT characteristics also have a significant impact regardless of how carbon emissions are measured. There is a clear association between the amount of Internet penetration in a certain industry and carbon emissions. Because of the G-7 economies ICT Masterplan, the provinces of G-7 countries have supported the adoption of ICT sector progress across the province, which may be the reason. The development of ICT infrastructure capable of supporting new environmentally friendly and efficient technologies is a key goal in this plan to encourage economic transformation. The estimated results are a counterpoint to prior studies that found ICT to be minor [81]. Furthermore, ICT has the potential to enhance human development, resulting in a manufacturing process that is focused on skills and is more ecologically sustainable [82]. In addition, the utilization of ICT has prompted economies to shift their reliance from physical resources to communication resources. This shift has resulted in reduced energy utilization and thus lower levels of CO_2_ emissions [83]. According to Zhu et al. [84], Green by ICT suggests that ICT can enhance the efficiency of various aspects of production, including design, manufacture, use, and end-of-life care. The optimization of individual components within product systems leads to enhanced energy efficiency across various sectors of the economy, hence facilitating energy conservation and the mitigation of carbon emissions.

The outcomes show that English Education (EE) positively influences ecological quality. CO_2_ emissions are positively correlated with level of education. In particular, it has been observed that education enhances the environmental condition of the G-7 countries. These results are consistent with recent investigations carried out by Li et al. [88]. The outcomes of our study show that the implementation of an environmentally appropriate curriculum is insufficient in mitigating CO_2_ emissions through education alone. Viable policy choices for promoting the environmental advantages of education include incorporating environmental content into educational materials, raising awareness through media channels, and providing energy efficiency training to the workforce. In order to fully capitalize on the advantages of education, it is imperative to establish a comprehensive framework of environmental protection legislation. Failure to do so would lead to a rise in individuals’ purchasing power, energy utilization, and consequently, potential harm to the environment. Investing in education enables a significant portion of the populace to enhance their understanding of their surroundings. Citizens that possess a heightened level of global consciousness are more inclined to adopt sustainable lifestyles. Consequently, the results obtained from panel-level and nation causality investigations predominantly support the theoretical expectations. Moreover, existing empirical studies have consistently demonstrated a significant influence of education on the environment [20,85]. In order to derive any advantages from education, it is imperative to establish a comprehensive framework of environmental protection legislation. Failure to do so would lead to an increase in individuals’ purchasing power, energy consumption, and thus, environmental degradation. The allocation of funds towards English Education (EE) enables a significant portion of the populace to enhance their understanding of their surroundings. Individuals who possess a heightened consciousness of global affairs are more inclined to adopt sustainable lifestyles. Consequently, the results obtained from panel-level and nation causality investigations predominantly support the theoretical expectations. Moreover, existing empirical studies have consistently demonstrated a substantial influence of education on the environment [86,87].

In addition, a correlation between carbon emissions and RE is negative, although minor. An upsurge in RE has a negligible influence on CO2 emissions under the AMG specification. In other words, policies that enhance social welfare and increase public knowledge of the benefits of renewable energy should be implemented. When this component rises by 1%, emissions fall by 0.12 percent [88]. This is consistent with previous relevant case studies. CO_2_ emissions, on contrary, fall as the amount of RE consumed grows. To put it another way, this study shows that increasing the percentage of RE usage does not significantly progress ecological quality. On the other hand, the expansion of RE usage increases CO_2_ emissions. A more accurate depiction of reality can be seen in the first case. As the share of RE utilization grows, it also means that fossil fuel consumption decreases significantly. In this scenario, it appears that growing the usage of RE can help meet global climate goals.

It is the final aspect of a green economy that has a negative impact on carbon emissions. CO_2_ emissions are reduced by 0.113 percent for every one percentage point increase. According to recent research, global air pollution and GHG emissions have been significantly reduced due to the COVID-19 pandemic’s lockdown measures [89–91]. In addition, they discovered that the ozone layer was improving and that various other factors, such as air and water quality, had improved as a result. There was no way for governments to continue lockdown measures for long periods of time so as to minimize the negative economic impact of COVID-19 infections. Even if the COVID-19 infection was still on the rise in 2020, a few governments eased their tight lockdown restrictions in whole or in part. Carbon emissions were not uniformly reduced by lockdown measures in the same country or different countries because of the differing types and lengths of lockdown measures enforced. Others implemented lockdowns across the country for several months in various cities or states, while others restricted movement for weeks or even months. As a result, although lockdown measures reduced carbon emissions, the global distribution of annual carbon emissions differed. According to the findings, carbon emissions were lower in highly impacted continents and more significant in less influenced continents. Lockdown measures’ strictness appeared to have a direct correlation with the infection rate and an inverse correlation with carbon emissions. On account of the severe influence of the COVID-19 on these regions’ annual carbon emissions, the countries of G-7 have imposed rigorous lockdown measures to halt the disease’s spread. Countries in the northwestern region of South America, Africa, and Australia were only marginally affected by the COVID-19 pandemic and did not impose stringent lockdown measures to limit the spread of the disease. In 2020, their annual carbon emissions will be greater. Earlier research, such as Dong et al. **[92]**, found that lockdown measures considerably reduced carbon emissions during short time periods (monthly to semi-annual). These new results complement those earlier studies. Overall, 2020 will see a decrease in carbon emissions and an increase in carbon uptake relative to previous years. Global declines in transportation (on land, water, and air), agricultural, and industrial production may be to blame, and Table 6 represents that the Outcomes of AMG Test.

**Table 6:** Outcomes of AMG test.

Variable	Coefficient	Std. Dev.	t-statistics	P-value
lnURB	00.6345***	1.2301	2.7563	1.000
lnGDPC	0.5401***	0.1319	4.0942	0.000
lnICT	-0.7321***	0.1376	-5.3215	0.005
lnEE	-0.6655***	0.1399	-4.7562	0.000
lnRE	-0.0124	0.0014	-9.1653	0.523
lnCovid-19	-0.1136***	0.0221	-5.1250	0.005
Cons.	3.1234***	1.6504	1.8925	0.001

Note: **, *** represents 5%, and 1% significance level, respectively.

The findings suggest that there is a positive relationship between GDP per capita, urbanization, and CO_2_ emissions in the G-7 economies. The data indicates that a one-unit increase in GDP per capita and urbanization is associated with a corresponding rise in CO_2_ emissions. Similarly, an increase of one unit in information and communication technology, English Education, energy from renewable sources usage, and Covid-19 would result in a reduction in carbon dioxide emissions in G-7 countries (See Table 7). Therefore, one could posit that a society characterized by a strong educational foundation is more likely to achieve sustainable economic growth [93]. The outcomes of our investigation align with the conclusions documented by Lim et al. [94]. Guth et al. [95] conducted a study that underscored the significance of education in facilitating the advancement of energy technologies with enhanced efficiency. The cultivation of human capital through education plays a crucial role in promoting equitable economic growth and development.

**Table 7:** Mediating effect results.

Variable	Coefficient	Std. Dev.	t-statistics	P-value
lnURB	0.3216**	0.1119	3.8736	0.042
lnGDPC	0.7653***	0.1664	4.5981	0.002
lnICT	-0.0906***	0.0165	-5.5142	0.000
lnEE	-0.5421**	0.5116	-1.0596	0.012
lnRE	-0.0752	0.0061	-12.3857	0.124
lnCovid-19	-0.2194**	0.0234	-9.3856	0.024
Ln(EE * ICT)	-0.6896**	0.1198	-5.7523	0.015
Cons.	1.6216***	0.4575	3.3957	0.005

Note: **, *** represents 5%, and 1% significance level, respectively.

### 4.2. D-H panel causality test

Table 8 illustrates the results of the D-H panel causality test, which provides strong evidence for two-way causality between all selected variables. The findings demonstrate the two-way causal Granger linkages between RGDP and emission. This panel’s economy can alter anytime, and pollution can affect economic growth. ED can be triggered by any change in this panel’s economic activities. Furthermore, economic progress and emission are closely linked, and these findings are consistent with [93–95]. Because of the bidirectional causality between RE and the economic institution’s performance, changes in biomass might have a significant impact on the environment. Likewise, a bi-directional causal association exists between urbanization and carbon emission. This concludes that any substantial change in the urban sector would cause a change in the carbon emission and vice versa. Also, the two-way causal association exists between internet users and the carbon emission, which infers that the policies relevant to the carbon emission and ICT are moving parallel with each other and cause to boot the level of the green and digital economy. In the last, the unidirectional causal relationship between Covid-19 and carbon emission. This explains that under the scenario of a pandemic, there found a decline the environmental pollution, which causes carbon emission. There is not any kind of evidence for the feedback hypothesis for carbon emission and Covid-19.

**Table 8:** Results of the D-H panel causality test.

Null hypothesis	W-stat	Zbar-stat	P-value
lnCO2 >> lnURB	2.6332	1.7886	0.005
lnURB >> lnCO2	6.2245	2.9645	0.000
lnCO2 >> lnGDPC	5.7425	6.2564	0.000
lnGDPC >> lnCO2	8.5962	5.1288	0.000
lnCO2 >> lnICT	9.4582	7.6652	0.002
lnICT >> lnCO2	5.2250	3.6523	0.000
lnCO2 >> lnEE	6.3466	5.2220	0.000
lnEE >> lnCO2	7.8800	4.3164	0.000
lnCO2 >> lnRE	10.502	8.2435	0.000
lnRE >> lnCO2	7.5869	53614	0.005
lnCO2 >> lnCovid-19	1.3265	0.5897	0.215
lnCovid-19 >> lnCO2	3.6235	2.8754	0.005

## 5. Conclusion and policy recommendation

In this paper, we first show the evolution of English education and internet uses on the national green economy in G-7 countries and investigate the drivers of the green economy for the selected panel using the STIRPAT model. So as to examine the planned objectives, AMG estimator is used in this study. The preservation of the environment is a pressing issue in today’s world, and experts have looked into a variety of potential threats to its quality. As urbanization has grown at an ever-increasing rate over the last few decades, it presents an enormous risk to the worldwide ecology. In addition to being a developing country, G-7 economies have a significant urbanization rate. The most important empirical conclusion indicates a connection between increased urbanization and increased carbon dioxide emissions that is statistically significant. Thus, we can say that urbanization in G-7 countries does not raise carbon emissions but reduces them, depriving the country’s green economy. Estimated results reveal that human capital and ICT both have a negative and significant influence on carbon dioxide emissions. Additionally, the data reveal that ICT reduces carbon emissions in education, industrial, residential, transportation, and other industries. In contrast, the impact of EE exhibits a similar trend. Research has demonstrated that English Education effectively reduces carbon dioxide emissions in the context of a pandemic. Furthermore, it is paradoxical that the Covid-19 outbreak leads to a drop-in pollution levels, resulting in an increase in per capita income. Additionally, the findings suggest that the combined effect of English Education and information and communication technology has a detrimental effect on carbon emissions.

### 5.1. Policy recommendations

This article posits that it is imperative for governments to prioritize sustainable urbanization as a means of safeguarding environmental quality. This can be achieved through the implementation of efficacious policies and strategies, as urbanization has been found to substantially augment CO_2_ emissions among G-7 nations. To ensure the environmental sustainability of urbanization, it is necessary to decrease the use of private vehicles through the improvement of public transportation initiatives, reduce industrial emissions by using energy-efficient technology, and integrate environmental strategies into the urbanization process. Proper planning and efficient designing can further mitigate the environmental impact of rapid urbanization by reducing energy consumption and transportation in metropolitan areas with well-planned infrastructure. The unplanned urbanization, as described in the aforementioned research, is a significant factor contributing to the adverse environmental effects of urbanization. The governments of G-7 countries must make concerted efforts and make gradual progress to mitigate its harmful influence on the environment. With the aim of mitigating the rapid population expansion, which is a significant factor contributing to urbanization; it is imperative to raise public awareness regarding birth control methods. Similarly, it is imperative to avert excessive urbanization by providing the rural populace with ample resources, hence obviating the necessity for them to relocate to metropolitan regions.

The outcomes of this study have led to several key policy recommendations. In metropolitan regions, greenhouse gases are a major source of CO_2_ emissions. Unfortunately, G-7 countries are seeing a rise in carbon emissions as a result of growing urbanization and overcrowding. In such a pandemic situation, policymakers and the government should put their attention on this issue and encourage urban development that is energy efficient as well as online purchasing. In order to prevent additional environmental degradation, long-term, logical urban planning must be implemented. It is also considerable to note that emissions from urban industrial regions have a negative influence on ecological quality; consequently, businesses should be motivated to implement energy-efficient and environmentally friendly technology practices. The government should step in and make it easier for businesses to switch to environmentally friendly practices. Fourth, urban tree planting will aid in absorbing CO_2_ emissions. Finally, the government should develop programs to educate the public about environmental degradation and preventive actions for ecological preservation with the support of educational institutions and other organizations/institutions, as well as through mass media. The findings possess significant policy consequences. In previous years, there has been a notable rise in the proliferation of colleges. However, it is imperative to prioritize the establishment of uniform standards and the enhancement of quality. The development of clean energy technology holds significant importance, particularly in the formulation of efficient energy policy. In the present setting, it is imperative for the state to promote and support the research and development endeavors of universities in order to foster the advancement of clean energy technologies. In addition, establishing a partnership between universities and industries can enhance technological advancements and expedite the incorporation of these innovations into the manufacturing process. As said by the findings of Mukherjee [96], there exists a disparity in environmental awareness between university students residing in urban areas and those residing in rural areas. Therefore, the expansion of English Education will enhance consciousness and safeguard environmental integrity. Moreover, the establishment of specialized departments focused on environmental protection and green energy technology inside universities, together with the expansion of the environmental portfolio, will result in a heightened demand for specialists proficient in identifying environmental challenges and formulating effective solutions. In a similar vein, the organization of seminars, conferences, and workshops by English Education institutions will serve as a significant catalyst in fostering comprehension and addressing environmental challenges.

However, the results show that economic expansion in G-7 economies are linked to negative externalities of environmental degradation, i.e., increased CO_2_ emissions into the atmosphere. In other words, the research shows that when a country’s economy grows, its environmental quality degrades due to rising carbon emissions. As a result, urbanization cannot be a determining factor for formulating measures to reduce environmental degradation in the country, and the government should take other issues into account instead. ICT has been shown to benefit the environment by improving environmental management and take part to dematerialization in a wide range of industrial sectors, which is consistent with earlier studies on the subject Developing ICT and English Education should be a priority for G-7 countries as they implement cooperative strategies to promote sustainable consumption and production. This suggests that G-7 economies should persist in enhancing and modernizing their ICT infrastructure in order to achieve the dual advantages of heightened economic productivity and diminished CO2 emissions. Given the region’s highly advanced ICT infrastructure, it is imperative to establish a policy framework that effectively utilizes ICT to mitigate environmental deterioration. It is notable that in countries with renewable energy sources, there has been a substantial expansion in ICT infrastructure, encompassing internet, broadband, and mobile phones. Consequently, there arises a must to ascertain the optimal deployment strategies for these technologies in order to mitigate environmental emissions that have adverse effects. The examination of consumption, production, and technical breakthroughs brought about by ICT should be undertaken by the governments of G-7 economies. In order to reduce environmental damage, it is imperative to ensure that the benefits of production and consumption are outweighed by advancements in science and technological improvements. In order to improve the quality of life through consumption and production, it is necessary to use technology and equipment that release emissions. In this context, research and development efforts should be directed towards the creation of low-carbon machinery, with the aim of mitigating CO2 emissions. As previously stated, while ICTs enhance societal well-being, they also contribute to global emissions by generating garbage, particularly from outdated equipment. Therefore, it is advisable to establish policies that provide guidance on the kind of products that may be imported, and in specific instances, to deter or prohibit their importation. The government of G-7 countries should prioritize the scrutiny of ICT devices and equipment utilized within their respective countries, as well as the energy sources employed to operate these devices and equipment. In recent decades, economic growth in the region has led to major environmental issues, as agriculture and industry are two of the region’s most important economic activities. As a result of these activities increasing demand for energy, which is currently dominated by fossil fuels, more carbon emissions may be produced. COVID-19 pandemic, on the other hand, can serve as a valuable lesson for governments and communities looking to reduce carbon emissions. The knowledge learned from the COVID-19 epidemic can also be used to implement efforts to reduce carbon emissions.

Throughout the data collection process, we encountered several difficulties related to the accessibility of pre-existing data, which constrained our ability to restrict the time frame. To enhance future study, we suggest that the information be partitioned into other subsets, specifically for estimating industrial, based, agriculture based, and service-based economies individually. This will yield more accurate conclusions and practical implications. Moreover, the variable of education can be categorized into elementary, secondary, and vocational education, so facilitating the formulation of precise educational policies aimed at achieving sustainable development. Furthermore, the analysis can be enhanced by include innovation, which aids in assessing the effectiveness of educational programs and the significance of a creative society in achieving sustainable economic growth and mitigating environmental risks. Future studies could go into a variety of different areas. This research assesses the impact of the ICT sector and English Education on carbon emissions. As a result, authorities should look at the effects of ICT at the industrial or even firm level. Investigating the influence of ICT on various Chinese industries and businesses. For example, the Internet has shattered the transport industry in the region by introducing a variety of new businesses. As a result, policymakers will better grasp how information and communications technology (ICT) impacts carbon emissions. No investigation was done into the length, degree, and type of lockdown measures enforced in the selected provinces and nations. Due to a lack of data, several provinces were not included in the study. Therefore, in its findings, this study does not consider other environmental metrics, such as ecological footprints. COVID-19-related activities have a significant impact on carbon emissions in China’s vegetation and partially vegetated areas, according to this study.

## Supporting information

S1 Data (XLSX)

## Abbreviations

ICT: Information & communication technology
EE: English Education
AMG: Augmented Mean Group
CO_2_: Carbon dioxide
SDG: Sustainable development goals
EKC: Environmental Kuznets Curve
GHG: greenhouse gas
EDU: Education
RE: renewable energy
URB: urbanization
GHG: greenhouse gas
